This article has been retracted.

# Effects of Obstructive Sleep Apnea-Hypopnea Syndrome and Cognitive Function in Ischemic Stroke Based on Linear Regression Equation

**DOI:** 10.1155/2022/4105169

**Published:** 2022-06-22

**Authors:** Peng Ji, Qixing Kou, Xueping Qu, Gen Sun, Songcan Liu, Jiewen Zhang

**Affiliations:** ^1^Zhengzhou University People's Hospital, Zhengzhou, Henan 450000, China; ^2^The Third People's Hospital of Zhengzhou (Tumor Hospital Affiliated of Henan University), Zhengzhou, Henan 450000, China

## Abstract

The objective of this research is to study the effect of obstructive sleep apnea-hypopnea syndrome on cognitive function of stroke. Based on linear regression equation and Montreal Cognitive Assessment Scale, the degree of cognitive impairment in OSAHS patients was evaluated and the influencing factors of OSAHS-induced cognitive impairment and the correlation between the degree of OSAHS and cognitive impairment were explored. The results are as follows: about 68% of OSAHS patients have cognitive dysfunction, and the incidence of cognitive dysfunction is positively correlated with OSAHS; cognitive impairment of OSAHS patients was associated with age, obesity, years of schooling, and intermittent nocturnal hypoxia or hypoventilation; the severity of cognitive dysfunction of OSAHS patients was positively correlated with age and obesity but negatively correlated with education level; Logistic regression analysis results showed that there were three factors that were finally entered into the regression equation, namely, LSaO2, BMI, and AHI, and the Logistic regression equation obtained was as follows: Logist*P* = −0.109*X*_1_ + 0.785*X*_2_ + 1.228*X*_3_. This study helps clinical workers to detect and intervene the impaired cognitive ability of patients with OSAHS early, so as to reduce the incidence and mortality of related complications and improve the quality of life of patients.

## 1. Introduction

In recent years, obstructive sleep apnea-hypopnea syndrome (OSAHS) is a kind of sleep disorder with serious harm to human health. Due to the complete or incomplete collapse and obstruction of the upper airway during sleep, apnea or hypopnea occurs repeatedly, causing indirect hypoxia hypercapnia and sleep structure disorder. The main clinical manifestations are snoring during sleep accompanied by recurrent apnea, daytime sleepiness, dry mouth, dizziness, headache, and fatigue, as shown in Figure 1 [1]. The incidence of OSAHS increases with age. For people under 70 years old, the risk of death will increase if risk factors such as obesity, smoking, and drinking are combined with OSAHS. At the same time, the investigation found that the incidence of OSAHS in males was higher than that in females. The incidence of OSAHS in adult males was 3%-7%, while that in adult females was 2%-5%. Moreover, the incidence of OSAHS in menopausal women was on the rise [2]. The differences in prevalence are due to regional and ethnic differences, age differences, and gender differences in epidemiological investigation methods. Due to the limitations of current epidemiological research methods, it is estimated that the actual prevalence of OSAHS should be higher than the above values. OSAHS is a disease involving multiple systems of the whole body, which can cause damage to multiple target organs of the whole body to a certain extent, such as cardiovascular and cerebrovascular diseases, diabetes, pulmonary heart disease, respiratory failure, and cognitive dysfunction. In recent years, studies have shown that the cognitive dysfunction caused by OSAHS patients is mainly mild cognitive impairment, and with the development of the disease, severe cases may evolve into Alzheimer's disease, among which the incidence of cognitive dysfunction is higher in severe OSAHS patients [3]. Stroke is a kind of cerebral blood circulation disorder with transient or permanent brain dysfunction as the main clinical manifestations. Acute ischemic stroke is a serious threat to patients' life safety due to its rapid onset and often without obvious prodromal symptoms. Studies have pointed out that sleep-disordered breathing is closely related to the prognosis of patients with cerebrovascular diseases, and the incidence of vascular dementia in patients with acute ischemic stroke complicated with OSAHS is significantly higher than that in patients without OSAHS [4]; therefore, it is of great significance to clarify the impact of OSAHS on patients with acute ischemic stroke and take targeted preventive measures to improve the prognosis of patients. Cognition refers to the ability of human brain to process, preserve, and extract information, which involves many fields such as learning, memory, execution, calculation, and understanding [5]. Cognitive dysfunction refers to the impairment of cognitive ability of different degrees caused by different factors. Clinically, it can be manifested as difficulty in concentration, memory decline, executive function decline, reasoning and abstract thinking ability decline, etc. There are more serious disorders such as agnosia and aphasia. At present, the clinical evaluation methods for the cognitive function of patients with OSAHS include the cognitive function assessment scale neuroelectrophysiological imaging. This study explored whether the cognitive function of patients with OSAHS is related to the severity of OSAHS. The objective of this research is to study the correlation between cognitive function and AHI LSaO2 ODI in patients with OSAHS.

## 2. Literature Review

Currently, the commonly used scales for cognitive function testing of OSAHS patients include Montreal Cognitive Assessment Scale (MoCA), Simple Mental State Examination Scale (MMSE), Wechsler Adult Intelligence Scale (WAIS), Extended Dementia Scale (ESD), Lowenstein Cognitive Scale Language Fluency Test (VFT), daily living activity scale, and complete neuropsychological test [6]. Because the assessment scale is relatively simple and time-consuming, it is widely used in the detection of cognitive function. WAIS is mainly aimed at the assessment of intelligence and operational ability, so it is not suitable to evaluate the neurological impairment of OSAHS patients alone. As the scale is complicated, it is also not suitable for large-sample tests. MMSE is widely used in the screening of cognitive dysfunction due to its strong sensitivity, easy operation, and less time-consuming. However, MMSE is relatively simple and easy to miss diagnosis of mild cognitive impairment [7]. ESD is a scale commonly used to assess brain cognitive function at home and abroad in recent years. Its content and items are more detailed, and it can reflect the brain cognitive function comprehensively and completely [8]. Some studies believe that MoCA is more reliable than MMSE in the detection of cognitive dysfunction in patients with OSAHS [9, 10].

Electroencephalography (EEG) and magnetoencephalography (MEG) are widely used in clinical neurophysiological examination [11]. It is believed that event-related potentials (ERPs) extracted from EEG and MEG are closely related to cognitive functions such as memory, judgment, and attention. The concept of event-related potentials was put forward, which provided a more objective and simple method for the study of cognitive function [12]. ERPs are the cognitive processing process of the human brain's perception of stimulus events and responses to stimulus events recorded on the tester's scalp surface, and the brain potentials are obtained by repeated superposition. It can be understood that it is the evoked potential of cognitive function. P300 is the main indicator for evaluating cognitive functions which are amplitude and latency. A cross-sectional study by Yang and Sun found poor differentiation of ERP waves in patients with cognitive dysfunction, the incubation period of P300 was prolonged, and the amplitude was significantly reduced. It can be used to assess whether a patient's cognitive function is impaired [13]. Compared with imaging, EPRs have the advantages of low cost, high time resolution, and noninvasive multimode assessment. It is a more objective, sensitive, and easy to operate electrophysiological technique for the assessment of cognitive dysfunction.

At present, the clinical evaluation methods for the cognitive function of patients with OSAHS include the Cognitive function Assessment Scale. The commonly used assessment scale for neuroelectrophysiological imaging is Montreal Cognitive Assessment (MoCA), Mini Mental Status Exam (MMSE), Expansive Scale of Dementia (ESD), etc. MMSE is too simple, insensitive to mild cognitive impairment, and ESD is complex and time-consuming, which is not suitable for the screening of cognitive impairment. Therefore, Montreal Cognitive Assessment Scale is commonly used to evaluate cognitive ability in clinical practice. Therefore, the Montreal Cognitive Assessment Scale (ERPs) is commonly used to evaluate the event-related potentials (ERPs) in neuroelectrophysiology of cognitive ability, in which P300 can be used to evaluate the impairment of cognitive function, which is relatively sensitive. Imaging is an objective and user-friendly assessment method, but it is rarely used in clinical assessment of cognitive function due to its radioactivity and high cost.

In recent years, more and more domestic and foreign scholars began to pay attention to and study the influencing factors and pathogenesis of cognitive dysfunction in OSAHS patients. Most scholars believe that the related factors affecting the cognitive dysfunction of OSAHS patients are as follows: education level, age, education level, obesity, smoking, nocturnal interrupted hypoxia, and sleep structure were considered to be the main factors. OSAHS patients have repeated intermittent hypoxia during sleep, which can lead to abnormal functional metabolism in the hippocampus and cerebellum and other areas of the brain and cause cognitive impairment in learning and memory behaviors. At the same time, hypoxia can produce a large number of oxygen free radicals and lead to oxidative damage, thus inducing neuronal apoptosis [14]. However, sleep fragmentation in OSAHS patients may cause changes in neurotransmitter concentration, resulting in impaired cognitive function. At present, the influencing factors and pathogenesis of cognitive dysfunction in OSAHS patients are still unclear, and there is a lack of large sample data studies, and there are also different literature reports at home and abroad [15].

Some studies believe that OSAHS patients have extensive cognitive dysfunction, which is positively correlated with the severity of OSAHS [16]. The main characteristic of the OSAHS patient is repeated intermittent hypoxia in the process of sleep, and hypoxemia can cause systemic dysfunction of many organs, among which the central nervous system is particularly sensitive to hypoxemia [17]. The hippocampal cerebellum and other structures of the brain are very sensitive to hypoxia, which can lead to abnormal brain function and metabolism in this region and cause cognitive impairment such as learning and memory behavior [18]. Morris water maze test was used to investigate the relationship between cognitive function and chronic intermittent hypoxia in rats. The results showed that the progressive decline of cognitive function in chronic intermittent hypoxia rats was associated with pathological injury of prefrontal cortex and hippocampal neurons and progressive reduction of ChAT expression. Studies have shown that the concentration and executive ability of patients with OSAHS are significantly decreased compared with normal people and are correlated with average blood oxygen saturation (*r* = −0.51, *P* = 0.002) and blood oxygen saturation < 90% (*r* = 0.56, *P* < 0.001), but not with daytime sleepiness. Recent studies have shown that chronic intermittent hypoxia can affect neuronal proliferation and differentiation, but there is no data to show whether chronic intermittent hypoxia increases or decreases neuronal proliferation [19]. Other studies suggest that chronic intermittent hypoxia may cause learning and memory impairment and increased apoptosis of hippocampal neurons through activation of Wnt/*β*-catenin, thus leading to cognitive dysfunction in OSAHS patients [20]. OSAHS patients repeatedly have apnea or hypoventilation at night, resulting in hypoxy-reoxygenation damage, resulting in increased oxide production and reduced antioxidant production, resulting in oxidation or antioxidant imbalance, and resulting in oxidative stress reaction [21, 22]. Oxidative stress can cause the release of various vasoactive substances and lead to vascular endothelial cell damage and endothelial dysfunction, resulting in atherosclerosis [23]. At the same time, hypoxemia can stimulate vasoconstriction and increase in red blood cells, which can cause slow blood flow of the body and then aggravate brain tissue ischemia and hypoxia, which in the long run causes extensive damage to brain cells and induces nerve cell apoptosis [24]. Neuronal apoptosis induced by cerebral ischemia and hypoxia is mainly located in the cerebral cortex and hippocampus, which are important parts of information processing, memory, and signal transmission [25]. Based on the current study, the Montreal Cognitive Function Assessment Scale was used to evaluate the cognitive function of the case group and the control group. The incidence of cognitive impairment in the case group with MoCA score of 26 as normal cognitive function (68%) was significantly higher than that in the control group (3%), and moderate to severe OSAHS was higher than that in mild OSAHS patients who are more likely to develop cognitive dysfunction. The detection rate of cognitive dysfunction is also different due to the difference of sample assessment methods and research methods.

## 3. Research Method

### 3.1. Research Object

A retrospective analysis was conducted on patients aged 18-70 years who complained of sleep snoring and daytime sleepiness in outpatient department of respiratory medicine or ward of a hospital from August 2021 to December 2021. All patients underwent PSG test and MoCA questionnaire for at least 7 hours overnight. During the examination, the subjects were not allowed to drink coffee or take sedative drugs.

### 3.2. Inclusion and Exclusion Criteria

Patients aged between 18 and 70 years old, with junior high school education or above, who could read and write Chinese, were included with the chief complaint of snoring during sleep and daytime sleepiness. The diseases related to cognitive impairment, such as frontotemporal lobe infarction, hypothyroidism, psychiatric diseases, or severe liver insufficiency with a history of psychiatric diseases, were excluded. Patients with history of drug abuse; with serious heart, liver, and kidney insufficiency or malignant tumor; complicated with pneumonia, asthma, chronic obstructive pulmonary disease, and other respiratory diseases; and with diabetes mellitus and vascular complications were excluded.

### 3.3. General Data Collection

A self-made questionnaire was used to collect general information of the subjects, including the following: gender, age, height, weight, occupation, education level, blood pressure, history of smoking and drinking, history of basic diseases such as cardiovascular diseases, history of brain trauma, and history of diabetes. BMI is calculated according to the height and weight. BMI = weight (kg) square (m^2^) of each height, BMI 24.0 is overweight, and BMI 28.0 is obese.

### 3.4. Cognitive Function Assessment

All subjects underwent MoCA to assess cognitive function. The MoCA scale includes the following: executive ability, naming, attention, speech, and other different cognitive areas. The total score of the scale is 30, and the score is 26, which is normal, and the higher the score is, the better the cognitive function is. Meanwhile, for ≤12 years of education, the MoCA score increases by 1 point.

### 3.5. Polysomnography (PSG)

All subjects underwent overnight PSG testing in a respiratory and sleep monitoring room of a hospital. Subjects were not allowed to use sedatives, alcohol, coffee, etc., within 24 hours before the examination. The monitoring time was from 22 : 00 p.m. to 7 : 00 p.m. the next day, and the monitoring content was mouth and nose airflow, chest respiration, pulse, oxygen, pulse, etc. Monitoring indicators include AHI, LSaO2, and ODI. All monitoring data are automatically analyzed by computer, and finally, the results are obtained after manual reading inspection and correction. Each AHI < 5 times was divided into control group, and each AHI < 5 times was divided into case group. The case group was divided into three groups (5 AHI 15 times per mild OSAHS, 15 < AHI 30 times per moderate OSAHS, and AHI 30 times per severe OSAHS).

### 3.6. Data Statistics and Analysis

A total of 128 patients were included in this study, including 32 in the control group and 32 in the case group with mild, moderate, and severe OSAHS. The SPSS20.0 statistical software was used to process the test data. The measurement data ± was expressed as mean standard deviation (*x* ± *s*), and the counting data was expressed as percentage, and pairwise comparison was used with*χ*^2^test. Logistic regression analysis was used to analyze the risk factors, and *P* < 0.05 was considered statistically significant.

## 4. Interpretation of Result

### 4.1. The General Situation of Case Group and Control Group

The average age of patients with mild, moderate, and severe OSAHS in the case group was 51.88 ± 10.59, 51.56 ± 10.99, and 43.34 ± 9.63, respectively; 15 (46.9%), 16 (50%), and 12 (37.5%) had high school education, 17 (53.1%), 16 (50%), and 20 (62.5%) had college education, and the average length of education was 13.84 ± 1.85, 13.72 ± 1.78, and 14.16 ± 1.74, respectively. Body mass indexes were (27.60 4.61) kg/m^2^, (27.40 3.13) kg/m^2^, and (29.12 3.66) kg/m^2^, respectively.

The average age of the control group was 45.78 ± 10.96. 11 (34.4%) have high school education, 21 (65.6%) have college education or above, and the average length of education is 14.25 ± 1.76. Body mass indexes were (26.13 3.99) kg/m^2^. There was no significant difference in the index of years of education among different groups (*P* = 0.593). The difference in BMI of age was statistically significant, as shown in Table 1.

### 4.2. The Incidence of Cognitive Dysfunction in Case Group and Control Group

In the case group, 65 patients showed cognitive impairment, i.e., MoCA score < 26, OSAHS with accounting for 68%. There were 11 cases (34 cases) in the mild OSAHS group. There were 25 cases (78%) in the moderate group. There were 29 cases (90%) in the severe group. One of the 32 control group had cognitive dysfunction. Chi-square test showed that the incidence of cognitive dysfunction was statistically different between the control group and the case group (*χ*^2^ = 62.436, *P* = 0.000), and the incidence of cognitive dysfunction in the non-OSAHS group was significantly lower than that in the OSAHS group. Meanwhile, the incidence of cognitive dysfunction in the moderate and severe OSAHS group was significantly higher than that in the mild OSAHS group, as shown in Table 2 and Figure 2.

### 4.3. Cognitive Impairment in Case Group and Control Group

In patients with mild to moderate OSAHS and the control group, MoCA scores from high to low were 27.72 ± 1.30, 26.03 ± 2.39, moderate, 24.63 ± 1.90, and 21.56 ± 3.23, respectively. The score difference was statistically significant (*F* = 40.609, *P* = 0.000). The moderate difference between the control group and OSAHS mild OSAHS was statistically significant (*P* ≤ 0.01). The moderate difference between the severe OSAHS group and the mild OSAHS group was statistically significant (*P* < 0.01), that is, the more severe the OSAHS patients were, the lower the MoCA score was. The language index of the control group was significantly different from that of the moderate OSAHS group (*P* ≤ 0.01). There was statistically significant difference between the mild OSAHS group and the moderate OSAHS group (*P* < 0.01). There was significant difference in delayed recall index between the control group and the moderate OSAHS group (*P* ≤ 0.01). There was statistically significant difference between the severe OSAHS group and the moderate OSAHS group (*P* < 0.01). There was significant difference in orientation index between the control group and the moderate OSAHS group (*P* ≤ 0.01). The difference between the severe OSAHS group and the mild OSAHS group was statistically significant (*P* < 0.05), as shown in Table 3 and Figures 3 and 4.

### 4.4. Logistic Regression Analysis of the Factors Affecting the Cognitive Function of OSAHS Patients

The cognitive function score of OSAHS patients was divided into a dichotomous variable by MoCA score of 26: (1) <26, indicating cognitive dysfunction and (2) a score of 26 indicates normal cognitive function. The dichotomies of cognitive function scores in the converted OSAHS group were used as dependent variables, and years of education, age, BMI, LSaO2, AHI, etc., were used as independent variables. According to the standard of *A* in = 0.05 *A* out = 0.10, a progressive binary Logistic regression analysis was performed to explore the age and years of education. The meanings and values of the variables influencing the cognitive function of patients with OSAHS, including BMI, LSaO2, and AHI, are shown in Table 4.

### 4.5. Multivariate Logistic Regression Analysis of Influence on Cognitive Function of Patients with OSAHS

The results of Logistic regression analysis showed that there were three factors that were finally entered into the regression equation, namely, LSaO2, BMI, and AHI, in which LSaO2 OR value and 95% CI were all <1, which were protective factors for the occurrence of cognitive dysfunction in OSAHS patients. The OR value and 95% CI of BMI and AHI were all >1, indicating that OSAHS is a risk factor for cognitive dysfunction in patients. With the increase of LSaO2, the risk of cognitive dysfunction in OSAHS patients decreased, and the OR value was 0.897 (95% CI: 0.815, 0.987). The increase of abnormal BMI also increased the risk of cognitive dysfunction in OSAHS patients, with an OR value of 2.133 (95% CI: 1.047, 4.346). Similarly, the increase of AHI anomaly level also increased the risk of cognitive dysfunction in OSAHS patients, and the OR value was 3.415 (95% CI: 1.695, 6.882), and the Logistic regression equation was Logist*P* = −0.109*X*_1_ + 0.785*X*_2_ + 1.228*X*_3_. The results of the multivariate logistic regression analysis are presented in Table 5.

## 5. Conclusion

About 68% of OSAHS patients showed cognitive impairment, and patients with moderate to severe OSAHS were more likely to develop cognitive impairment than those with mild OSAHS. Cognitive dysfunction of OSAHS patients was associated with age, obesity, education, and intermittent nocturnal hypoxia or hypoventilation. Age, obesity, and education level are risk factors for cognitive dysfunction in OSAHS patients. The severity of cognitive dysfunction of OSAHS patients was positively correlated with age and obesity and negatively correlated with education level. The results of this study showed that the total MoCA score of OSAHS patients was negatively correlated with AHI and positively correlated with the lowest blood oxygen saturation at night. The orientation of visual spatial attention language delay recall was negatively correlated with AHI. Delayed recall of visuospatial attention language was positively correlated with the lowest blood oxygen saturation at night. The results showed that patients with more severe nocturnal hypoxia or hypoventilation had more severe cognitive impairment, especially in visual spatial attention, language delay, recall orientation, and other aspects, confirming that nocturnal hypoxia or hypoventilation is one of the influencing factors of cognitive function in patients with OSAHS. However, whether nocturnal hypoxia or hypoventilation causes cognitive dysfunction in OSAHS patients through oxidative stress inflammatory response or apoptosis induction needs further research and exploration. The older the age, the higher the BMI, and the more severe the cognitive dysfunction. At the same time, the more times of nocturnal apnea and hypopnea in OSAHS patients, the lower the minimum blood oxygen saturation at night, and the more serious the cognitive function impairment, especially in memory, attention, and language.

## Figures and Tables

**Figure 1:** Obstructive sleep apnea-hypopnea syndrome.

**Figure 2:** MoCA score of the case group and control group. Note: the total score of MoCA was 30, and 26 was normal.

**Figure 3:** Visual spatial score of the case group and control group. Note: the total score of visual space is 5.

**Figure 4:** Delayed recall scores in the case group and control group. Note: the total score of delayed recall was 5.

**Table 1:** Comparison of general situation between the case group and the control group.

Project	Control group	OSAHS mild	OSAHS moderate	OSAHS severe	*F*	*P*
Age (years)	45.78 ± 10.96	51.88 ± 10.59^b^	51.56 ± 10.99^a^	43.34 ± 9.63	5.190	0.002
Years of education (years)	14.25 ± 1.76	13.84 ± 1.85	13.72 ± 1.78	14.16 ± 1.74	0.637	0.593
BMI	26.13 ± 3.99^a^	27.60 ± 4.61	27.40 ± 3.13	29.12 ± 3.66	3.183	0.026

Note: compared with the OSAHS severe group, ^a^*P* < 0.05 and ^b^*P* < 0.01.

**Table 2:** Comparison of the incidence of cognitive dysfunction between the case group and the control group.

Grouping	Cognitive function		*χ* ^2^	*P*
	Normal	Abnormal		
Control group	31	1		
OSAHS mild	21	11		
OSAHS moderate	7	25	62.436	0.000
OSAHS severe	3	29		
Add up	62	66		

**Table 3:** Cognitive impairment in case group and control group.

Project	Control group	OSAHS mild	OSAHS moderate	OSAHS severe	*F*	*P*
MoCA grade	27.72 ± 1.30	26.03 ± 2.394^a^	24.63 ± 1.90^a^	21.56 ± 3.23^bc^	40.609	0.000
View space	4.75 ± 0.44	4.38 ± 0.98	4.56 ± 0.76	3.72 ± 1.17^ac^	8.339	0.000
Name	2.91 ± 0.3	2.78 ± 0.55	2.88 ± 0.42	2.94 ± 0.25	0.924	0.431
Notice	5.75 ± 0.44	5.5 ± 0.57	4.81 ± 0.74^ab^	4.66 ± 1.07^ab^	16.252	0.000
Language	2.09 ± 0.64	2.06 ± 0.76	1.41 ± 0.5^ab^	1.5 ± 0.62^ab^	10.398	0.000
Abstract	1.94 ± 0.25	1.72 ± 0.52	1.78 ± 0.49	1.59 ± 0.67	2.571	0.057
Delayed recall	4.00 ± 0.149	3.28 ± 0.239	3.09 ± 0.231^a^	1.44 ± 0.25^abc^	24.119	0.000
Directive force	5.97 ± 0.18	5.81 ± 0.4	5.53 ± 0.72^a^	5.38 ± 0.71^ad^	7.650	0.000

Note: compared with the control group, ^a^*P* ≤ 0.01; compared with the mild group, ^b^*P* < 0.01; compared with the moderate group, ^c^*P* < 0.01; compared with the mild group, ^d^*P* < 0.05.

**Table 4:** Logistic regression analysis variable meaning and assignment description.

*Y* (MoCA total marks)	Normal (≥26 marks) = 0, abnormal (<26 marks) = 1
*X*_2_ (age)	<40 years = 1 = *X*_21_, 40 − 49 years = 2 = *X*_22_, 50 − 59 years = 3 = *X*_23_, ≥60 years = 4 = *X*_24_
*X*_3_ (education years)	≤9 years = 1 = *X*_31_, 10 − 12 years = 2 = *X*_32_, ≥13 years = 3 = *X*_33_
*X*_4_ (BMI)	Normal (18.5‐23.9) = 2 = *X*_41_, overweight (24.0‐27.9) = 2 = *X*_42_, obesity (≥28) = 3 = *X*_43_
*X*_5_ (apnea and hypopnea index)	Normal (<5 times/h) = 1, mild (5‐15 times/h) = 2 Moderate (15 − 30 times/h) = 3, severe (>30 times/h) = 4
*X*_6_ (minimum oxygen saturation at night)	Normal (>90%) = 1, mild (85%‐90%) = 2 Moderate (80% − <85%) = 3, severe (<80%) = 4

**Table 5:** Logistic regression analysis results.

	Regression coefficient	Standard error	Wald	*P*	OR	95% CI of OR	
Minimum sATS (*X*_6_)	-0.109	0.049	4.965	0.026	0.897	0.815	0.987
BMI (*X*_4_)	0.758	0.363	4.357	0.037	2.133	1.047	4.346
AHI (*X*_5_)	1.228	0.357	11.806	0.001	3.415	1.695	6.882

## Data Availability

The data used to support the findings of this study are available from the corresponding author upon request.
